The article "Three Mediating Pathways of Anxiety and Security in the Relationship between Coping Style and Disordered Eating Behaviors among Chinese Female College Students" was retracted in 2023. Reasons: signs of a paper mill; suspected computer-generated content; unreliable results or conclusions; lack of ethics approval or compliance.

# Three Mediating Pathways of Anxiety and Security in the Relationship between Coping Style and Disordered Eating Behaviors among Chinese Female College Students

**DOI:** 10.1155/2021/7506754

**Published:** 2021-09-20

**Authors:** Wenyue Han, Zheng Zheng, Ning Zhang

**Affiliations:** ^1^School of Medicine & Holistic Integrative Medicine, Nanjing University of Chinese Medicine, Nanjing, China 210023; ^2^Nanjing Brain Hospital Affiliated to Nanjing Medical University, Nanjing, China 210029

## Abstract

**Background:**

According to previous studies, eating disorders and disordered eating behaviors are associated with coping style, anxiety, and sense of security. However, the specific mechanism between them has not been elucidated. The purpose of this study was to explore whether anxiety and sense of security play mediating roles in coping style and disordered eating behaviors among Chinese female college students.

**Method:**

Six hundred and ninety-one female college students (mean age = 19.36; SD = 1.06) completed the Simple Coping Style Questionnaire, the Eating Disorder Inventory, the Security Questionnaire, the Hospital Anxiety and Depression Scale, and a brief demographic survey. The percentage bootstrap method of deviation correction was conducted to determine the mediating effect of anxiety and sense of security on coping style and disordered eating behaviors.

**Results:**

Coping style had direct and indirect effects on disordered eating behaviors. Anxiety and sense of security were not only independent mediators in the relationship between coping style and disordered eating behaviors but also chain mediators.

**Conclusions:**

The results of the current study provide preliminary evidence that preventive interventions targeting anxiety and sense of security may be feasible for young women who develop disordered eating behaviors due to stress in their lives.

## 1. Introduction

Eating disorders are prevalent, severe psychiatric disorders and often emerge during college-age women [1, 2]. Ward and his colleagues found that the incidence of eating disorders peaked at age 21, with initial onset mostly before the age of 25 [3]. Before meeting an eating disorder diagnosis, these young women often exhibit varying degrees of disordered eating behaviors, including overeating and restricted eating [4].

It has been reported that eating disorders and disordered eating behaviors are related to coping style and anxiety. Coping style reflects an individual's attitude and behavior pattern when facing various events in life. Anxiety is the most common comorbid diagnose in eating disorders [5]. Studies have shown that negative coping style is remarkably correlated with bulimia [6] and high anxiety level [7]. In addition, if individuals adopt positive coping style, they will have lower anxiety level and healthier eating behaviors [8–10].

The article "Three Mediating Pathways of Anxiety and Security in the Relationship between Coping Style and Disordered Eating Behaviors among Chinese Female College Students" was retracted in 2023. Reasons: signs of a paper mill; suspected computer-generated content; unreliable results or conclusions; lack of ethics approval or compliance.

Other studies have examined the relationship between coping style, sense of security, and eating behaviors. Sense of security refers to the perception of potential psychological and physiological risks, as well as the individual's self-efficacy in risk management, which is generally manifested as interpersonal security and certainty of control [11]. Individuals with negative coping style tend to have lower sense of security and higher social anxiety [12]. Uncertainty caused by insecurity reduces people's ability to control themselves and leads to overeating [13]. Moreover, the negative coping style of individuals with low sense of security prevents them from acquiring necessary social skills, which leads to interpersonal stress and further disordered eating behaviors [14].

Based on these studies, coping style, anxiety, sense of security, and disordered eating behaviors are related. However, no study has studied all four variables simultaneously to explore the specific mechanism between them. Therefore, this study will verify the specific role of anxiety and sense of security in coping style and disordered eating behaviors and provide theoretical basis for early intervention of disordered eating behaviors and prevention of eating disorders. We hypothesized that coping style not only directly affects disorder eating behaviors but also indirectly influences disordered eating behaviors through the mediating role of anxiety and sense of security.

## 2. Methods

### 2.1. Participants

The study sample comprised 691 female college students in Eastern China. Demographic characteristics of the sample are summarized in Table 1.

### 2.2. Measures

#### 2.2.1. Demographic Questionnaire

Participants completed a demographic questionnaire constructed to gather information about their age, hometown, and major.

#### 2.2.2. Disordered Eating Behavior

The Eating Disorder Inventory (EDI) is a 64-item self-report inventory consisting of 8 subscales: (1) drive for thinness, (2) body dissatisfaction, (3) bulimia, (4) perfectionism, (5) interpersonal distrust, (6) mature fear, (7) interoceptive awareness, and (8) inefficiency. The questions are presented on a six-point Likert scale, with scores ranging from 0 to 5 for each disordered eating behavior. The 8 subscales are calculated by totaling the items on each respective scale, while the total EDI score is calculated by adding all items together. Higher total EDI scores indicate more severe disordered eating behaviors [15]. In the current study, internal consistency *α* = 0.903.

The article "Three Mediating Pathways of Anxiety and Security in the Relationship between Coping Style and Disordered Eating Behaviors among Chinese Female College Students" was retracted in 2023. Reasons: signs of a paper mill; suspected computer-generated content; unreliable results or conclusions; lack of ethics approval or compliance.

#### 2.2.3. Coping Style

The Simple Coping Style Questionnaire (SCSQ) contains 20 items which effectively reflect the individual's coping style in the context of Chinese culture. Items 1-12 belong to positive coping and 13-20 belong to negative coping. The score of each item is from 0 (never) to 3 (always). If the Z score difference between positive coping and negative coping is greater than 0, it is positive coping; if less than 0, it is negative coping [16]. In the present study, total questionnaire internal consistency *α* = 0.77.

#### 2.2.4. Sense of Security

The Security Questionnaire (SQ) consists of 16 items, including 2 subscales of interpersonal security (personal security experience in interpersonal communication) and certainty of control (personal life prediction, sense of certainty and control). Each subscale has 8 items, and the score of each item is from 1 (not consistent at all) to 5 (completely consistent). Higher total SQ scores indicate higher sense of security [11]. In the current study, internal consistency *α* = 0.89.

#### 2.2.5. Anxiety

The Hospital Anxiety and Depression Scale (HAD) is a 14-item self-rating scale that measures symptoms of anxiety and depression respectively. Each item is scored from 0 to 3. The overall score for depression or anxiety can be considered the severity of the symptoms. The anxiety subscale has 7 items, and higher total scores indicate higher level of anxiety [17]. The internal consistency of this study *α* = 0.81.

### 2.3. Procedures

Participants were recruited through psychological health classes. Assessments took place in class and were supervised by members of the research team. The survey lasted half an hour, and questionnaires were collected on the spot. The effective recovery rate of the questionnaires was 97.3%. The research was approved by the Human Research Ethics Committee of NJUCM. Study information was provided directly to participants and informed consent was obtained.

### 2.4. Statistical Analysis

Analyses were performed using SPSS22.0. All statistical tests were two-tailed, and the significance level was set at *p* < 0.05. Pearson's correlation was used to examine the correlations between coping style, disordered eating behaviors, anxiety level, and sense of security. *T*-test was used to analyze the effects of coping style on anxiety, sense of security, and disordered eating behaviors. The mediation model was examined by PROCESS program developed by Preacher and Hayes [18], and the percentage bootstrap method of deviation correction was used to test the significance of mediating effect [19].

### 2.5. Common Method Biases

The Harman single-factor test was used to eliminate the common method deviation caused by the questionnaire survey. The results of factor analysis showed that the characteristic roots of 26 factors were greater than 1, and the explained variance percentage of the first common factor was 13.63% (less than 40%), indicating that there was no obvious method error.

The article "Three Mediating Pathways of Anxiety and Security in the Relationship between Coping Style and Disordered Eating Behaviors among Chinese Female College Students" was retracted in 2023. Reasons: signs of a paper mill; suspected computer-generated content; unreliable results or conclusions; lack of ethics approval or compliance.

## 3. Results

### 3.1. Correlations between Coping Style, Anxiety, Sense of Security, and Disordered Eating Behaviors

As shown in Table 2, coping style was negatively correlated with anxiety and disordered eating behaviors (*r* = −0.418, -0.318, *p* < 0.001) and was positively correlated with sense of security (*r* = 0.510, *p* < 0.001). Sense of security was negatively correlated with anxiety and disordered eating behaviors (*r* = −0.551, -0.414, *p* < 0.001). Anxiety was positively correlated with disordered eating behaviors (*r* = 0.443, *p* < 0.001).

### 3.2. Effects of Coping Style on Anxiety, Sense of Security, and Disordered Eating Behaviors

According to the score of SCSQ, the participants were divided into positive or negative coping style. As illustrated in Table 3, there were significant differences in disordered eating behaviors, sense of security, and anxiety between positive and negative coping styles (*t* (1,689) = −6.36, 11.33, -9.07; *p* < 0.001).

### 3.3. Mediating Effect Test

Table 4 revealed that coping style had a direct negative predictive effect on anxiety (*β* = −0.310, *p* < 0.001) and a direct positive predictive effect on sense of security (*β* = 0.250, *p* < 0.001). Anxiety had a direct negative predictive effect on sense of security (*β* = −0.408, *p* < 0.001). When coping style, anxiety, and sense of security predicted disordered eating behaviors simultaneously, coping style and sense of security had negative predictive effects (*β* = −0.067, -0.207; *p* < 0.05, 0.001), and anxiety had a positive predictive effect (*β* = 0.290, *p* < 0.001).

As shown in Table 5, analyses of total indirect effects indicated that anxiety and sense of security partially mediated the relationship between coping style and disordered eating behaviors (Effect = −0.168, SE = 0.020, 95% CI (-0.208, -0.131)). The mediating effect accounted for 71.8% of the total effect (Effect = −0.234, SE = 0.027, 95% CI (-0.287, -0.182)). In the meantime, when tested separately, three mediating paths were significant: coping style ⟶ anxiety ⟶ disordered eating behaviors (Effect = −0.090, SE = 0.020, 95% CI (-0.131, -0.053)), accounting for 38.5% of the total effect; coping style ⟶ sense of security ⟶ disordered eating behaviors (Effect = −0.052, SE = 0.160, 95% CI (-0.084, -0.022)), accounting for 22.2% of the total effect, and coping style ⟶ anxiety ⟶ sense of security ⟶ disordered eating behaviors (Effect = −0.026, SE = 0.087, 95% CI (-0.044, -0.010)), accounting for 11.1% of the total effect. The specific paths are presented in Figure 1.

The article "Three Mediating Pathways of Anxiety and Security in the Relationship between Coping Style and Disordered Eating Behaviors among Chinese Female College Students" was retracted in 2023. Reasons: signs of a paper mill; suspected computer-generated content; unreliable results or conclusions; lack of ethics approval or compliance.

## 4. Discussion

The purpose of this study was to explore whether anxiety and sense of security play mediating roles in coping style and disordered eating behaviors among Chinese female college students. To the best of our knowledge, this is the first empirical study to evaluate these relationships in a sample of female women. Our study found that, first of all, coping style was negatively correlated with anxiety and disordered eating behaviors while positively correlated with sense of security. And there were significant differences in anxiety, sense of security, and disordered eating behaviors between positive coping style and negative coping style. These results correspond to previous research findings, which have indicated negative coping style could lead to more severe disordered eating behaviors [20], higher level of anxiety [21], and lower sense of security [22]. Next, when analyzing the mediating roles of anxiety and sense of security between coping style and disordered eating behaviors, we found an overall mediating role of 71.8%. These results revealed that coping style had both direct and indirect effects on disordered eating behaviors. Through further analysis, we found three indirect effect pathways. The first pathway was coping style ⟶ anxiety ⟶ disordered eating behaviors, which indicated that negative coping style could enhance anxiety level and further induced more serious disordered eating behaviors. The second pathway was coping style ⟶ sense of security ⟶ disordered eating behaviors, which showed that negative coping style could reduce the sense of security and led to the aggravation of eating problems. Similar findings have been observed in previous studies [23, 24]. The third pathway was coping style ⟶ anxiety ⟶ sense of security ⟶ disordered eating behaviors, which illustrated that anxiety and sense of security played a chain mediating role in the relationship between coping style and disordered eating behaviors. In other words, negative coping style enhanced anxiety level, high anxiety level reduced the sense of security, and further aggravated disordered eating behaviors. Kuipers and his colleagues have found that when the symptoms of eating disorders alleviated, patients' anxiety and sensitivity to others were reduced, and their ability to deal with new situations was enhanced [25], which well supports the existence of chain mediating role identified in our study.

Findings from the present study have clinical implications for psychologists who work with young women. The present study provides evidence that negative coping style leads to higher anxiety level, lower sense of security, and more severe disordered eating behaviors. These findings provide preliminary support for targeting anxiety and sense of security in preventative interventions, particularly for female youth that have the propensity to disordered eating behaviors in response to feelings of stressful daily life. In clinical interventions, while therapists could help clients with eating disorders or disordered eating behaviors by teaching them coping strategies, the improvement of coping skills requires long-term learning and practice. In contrast, the regulation of anxiety is flexible and diversified, such as progressive muscle relaxation, meditation, breathing exercises, and visualization [26]. Therefore, if therapists aim at anxiety, they might achieve ideal effect in reducing disordered eating behaviors in a short period of time. In addition, due to the existence of chain mediating role, reducing anxiety also helps to improve safety and further alleviate disordered eating behaviors.

The article "Three Mediating Pathways of Anxiety and Security in the Relationship between Coping Style and Disordered Eating Behaviors among Chinese Female College Students" was retracted in 2023. Reasons: signs of a paper mill; suspected computer-generated content; unreliable results or conclusions; lack of ethics approval or compliance.

There are several limitations to the present study. Considering the present sample was restricted to female college students in East China, the findings may have limited generality. Besides that, the cross-sectional nature of this study prevents us from inferring causation. Future longitudinal studies are necessary to examine what predictive roles anxiety and sense of security play in mediating the relationship between negative coping style and disordered eating behaviors in female youth.

## Figures and Tables

**Figure 1:** Model of mediating roles of anxiety and sense of security between coping style and disordered eating behaviors.

**Table 1:** Demographic characteristics of study participants.

Characteristic	*N* or mean	% or SD	Range
Age (years)	19.36	1.06	18-22
Hometown			
Urban area	429	62.1%	
Rural area	262	37.9%	
Major			
Science and engineering	141	20.4%	
Medicine	273	39.5%	
Art	80	11.6%	
Liberal arts	197	28.5%	
Eating Disorder Inventory (EDI)			
Drive for thinness	4.49	4.54	0-21
Body dissatisfaction	10.65	6.45	0-27
Bulimia	1.97	2.87	0-21
Perfectionism	4.91	3.51	0-18
Interpersonal distrust	3.38	3.10	0-21
Mature fear	7.72	4.32	0-24
Interceptive awareness	4.21	4.34	0-27
Inefficiency	4.17	3.99	0-23
Total	41.50	20.69	4-139
Simple Coping Style Questionnaire (SCSQ)			
Positive coping style	350	50.65%	
Negative coping style	341	49.35%	
Security Questionnaire (SQ)			
Interpersonal security	27.33	5.35	8-40
Certainty of control	25.96	5.68	8-40
Total	53.29	10.30	16-80
Hospital Anxiety and Depression Scale (HADS)			
Anxiety	6.71	3.09	0-19

The article "Three Mediating Pathways of Anxiety and Security in the Relationship between Coping Style and Disordered Eating Behaviors among Chinese Female College Students" was retracted in 2023. Reasons: signs of a paper mill; suspected computer-generated content; unreliable results or conclusions; lack of ethics approval or compliance.

**Table 2:** Correlations between coping style, anxiety, sense of security, and disordered eating behaviors.

	1	2	3	4
(1) Coping style	1			
(2) Anxiety	-0.418^∗∗∗^	1		
(3) Sense of security	0.510^∗∗∗^	-0.551^∗∗∗^	1	
(4) Disordered eating behaviors	-0.318^∗∗∗^	0.443^∗∗∗^	-0.414^∗∗∗^	1

^∗∗∗^*p* < 0.001 (two-tailed), ^∗∗^*p* < 0.01 (two-tailed), and ^∗^*p* < 0.05 (two-tailed).

**Table 3:** Effects of coping style on anxiety, sense of security, and disordered eating behaviors.

	Positive coping style (*n* = 350)	Negative coping style (*n* = 341)	*t*
Disordered eating behaviors	36.71 ± 18.27	46.48 ± 21.86	-6.36^∗∗∗^
Sense of security	57.33 ± 8.76	49.16 ± 10.13	11.33^∗∗∗^
Anxiety	5.72 ± 2.66	7.74 ± 3.17	-9.07^∗∗∗^

^∗∗∗^*p* < 0.001 (two-tailed), ^∗∗^*p* < 0.01 (two-tailed), and ^∗^*p* < 0.05 (two-tailed).

**Table 4:** Regression analysis between variables.

Regression equation		Global fit index			Significance of regression coefficient	
Outcome variable	Predictor variable	*R*	*R* ^2^	*F*	*β*	*t*
Anxiety	Coping style	0.418	0.175	145.642	-0.310	-12.068^∗∗∗^
Sense of security	Coping style	0.631	0.399	228.112	0.250	10.409^∗∗∗^
	Anxiety				-0.408	-12.598^∗∗∗^
Disordered eating behaviors	Coping style	0.494	0.244	73.756	-0.067	-2.306^∗^
	Anxiety				0.290	7.194^∗∗∗^
	Security				-0.207	-4.835^∗∗∗^

^∗∗∗^*p* < 0.001 (two-tailed), ^∗∗^*p* < 0.01 (two-tailed), and ^∗^*p* < 0.05 (two-tailed).

**Table 5:** The mediating effect of anxiety and security between coping style and disordered eating behaviors.

	Effect value	Boot SE	Boot CI lower	Boot CI upper	Relative mediation effect
Total effect	-0.234	0.027	-0.287	-0.182	100%
Total indirect effect	-0.168	0.020	-0.208	-0.131	71.8%
Indirect path 1	-0.090	0.020	-0.131	-0.053	38.5%
Indirect path 2	-0.052	0.160	-0.084	-0.022	22.2%
Indirect path 3	-0.026	0.087	-0.044	-0.010	11.1%

Indirect path 1: coping style ⟶ anxiety ⟶ disordered eating behaviors; Indirect path 2: coping style ⟶ sense of security ⟶ disordered eating behaviors; Indirect path 3: coping style ⟶ anxiety ⟶ sense of security ⟶ disordered eating behaviors.

## Data Availability

Data and questionnaires are available upon request, contact at zzdoctor@126.com.
